# Green Financial Health Risk Early Monitoring of Commercial Banks Based on Neural Network Model in a Small Sample Environment

**DOI:** 10.1155/2022/4613088

**Published:** 2022-09-22

**Authors:** Shaohuang Wang

**Affiliations:** Cardiff University, Cardiff CF10 3AT, UK

## Abstract

Financial innovations emerge in an endless stream, and it is difficult for the regulatory measures and efforts of banks in various countries and the credit risk management level of commercial banks themselves to adapt to the increasingly complex risk environment faced by banks. In the process of building GFR (green financial risk) mixed governance model, the division of powers and responsibilities of governance subjects should be effectively defined. Therefore, it is very necessary to comprehensively and systematically study and grasp the characteristics, performance, and causes of commercial banks' GFR and build an early-warning model of commercial banks' GFR to comprehensively monitor the risks of banks, so as to reduce risks and avoid crises. Therefore, this paper uses the forward three-layer BPNN (BP neural network) technology to establish a real-time warning model of commercial banks' GFR. IL (input layer) to HL (hidden layer) adopts Sigmoid function, while HL to OL (output layer) function adopts linear function Purelin function. The results show that the test result of this method is greatly improved compared with the traditional method, and the correct rate is increased from 81.27% to 94.38%. It shows that the model in this paper has achieved a good warning effect of GFR for commercial banks.

## 1. Introduction

Different from traditional finance, which focuses on the theory and practice of money and banking, environmental finance takes the limited environmental capacity as the premise, links environmental issues with financial activities, and emphasizes paying attention to and realizing environmental sustainable development with financial instruments. The main reason for the decline of green financial resource allocation efficiency is that government departments, financial institutions, and enterprises have not made a reasonable assessment of the positive externalities of green industries in the field of environmental protection, which leads to incorrect prejudgment and finally improves the profit-seeking of capital [1]. The development of green finance has been supported by policies and guaranteed in terms of talents, materials, and technology [2]. We can see that green finance has formed a concept and spirit in developed countries, and at the same time, they have been refined into specific regulations and index systems, which have been truly implemented and continuously improved. The social benefits of green financial eco-environmental protection project investment are obvious, but the benefits and risks are uncertain. Therefore, the macro-prudential supervision standard of green financial projects is not high, and there are many loopholes in micro-prudential supervision, which is also the key factor to form the risk of green financial practice.

The conversion of the traditional financial sector to the green financial sector may face difficulties in the short term, including rising costs for new mechanisms and an increase in customer numbers. This will have a short-term negative impact on the sector's interests. On the other hand, long-term repercussions of traditional finance industry's non-“greening” economic operations can be mitigated by the development of new financial instruments, such as “green credit.” The role of finance in economic growth must be sustainable [3]. Financial innovations come out in a never-ending stream, making it difficult for banks in different countries to adapt their regulatory measures and efforts to the increasingly complicated risk environment that banks must deal with, as well as their own degree of credit risk management. While few studies have been done on the GFR (green financial risk) system and commercial bank risk supervision, all reputable organisations and academics are primarily focused on researching online banking acceptance models and risks. Credit risk has many adverse effects on the healthy development of state-owned commercial banks. Because commercial banks need to consume a lot of profits to extract and write off bad debts, it is difficult to effectively supplement their capital. Therefore, we should study how environmental protection and finance can be better integrated to form green finance; What projects should green finance serve?

From the policy environment of green financial development, although the state strongly advocates green environmental protection industry and gives support and inclination in policy, there is no coordination mechanism and implementation mechanism with high synergy among the industrial policies of related departments, the industrial policies of financial institutions and the financial policies of local governments. In the process of constructing GFR mixed governance model, the division of powers and responsibilities of governance subjects should be effectively defined. Because green finance is just emerging, it is still a new financial method, which is unstable in many aspects, especially the research on risk is relatively simple, so it is imperative to develop its risk early warning research. In view of the current situation that GFR early warning is not perfect at home and abroad, a new GFR early warning model of commercial banks is established by using neural network model. According to the reliable data of various indicators of the system, the current development of green finance of commercial banks is analyzed, and constructive suggestions are put forward according to local conditions. The main contributions of this paper are as follows: (1) the important part of the model input is the index system. In the research, the input index is divided scientifically and reasonably, and a comprehensive index system is concluded and established, which can correct the index in time clearly and ensure the dynamic adaptability of the whole model. (2) Green finance is still unexplored in the research and analysis of commercial banks' GFR early warning system because it is a relatively new business strategy. The model is more trustworthy when BPNN is used to test it, which is also novel for risk warning.

## 2. Related Work

### 2.1. Research on Financial Early Warning

GFR has a two-way effect. Among them, the function of the risk hazard ecological protection project can effectively reduce the performance level of ecological construction and protection management and cannot solve the harm caused by the ecological environment crisis to the public from the root cause, while financial institutions should be self-reliant and actively build a virtuous cycle of external regulation system and endogenous supervision system.

Early warning means warning in advance, reminding people to pay attention to the unbalanced state, abrupt events, and disordered structure that will appear in the operation of the system, so as to take timely measures to push the system to a new structural state. Financial early warning is the result of applying the idea of early warning to the financial field. Zhu and Liu used statistical methods to select evaluation indexes and give them weights. In the inspection report data, they calculated index scores and comprehensive scores, and according to the comprehensive scores, they rated the level of individual financial institutions [4]. Wang and Xie think that in an early warning system, an early warning sample is a pattern, and all samples with the same alarm degree form a class [5]. Rachmawati et al. think that although the design of probabilistic pattern classification early warning system needs prior probability, conditional probability or posterior probability, pattern recognition has provided many theoretical methods, which can solve many difficulties in the practical application of early warning [6].

The financial hazards of banks were examined by Li et al. using multiple discriminant analysis. It is noted that the discriminant function prediction will be more accurate the closer the time to the actual occurrence of business risks for commercial banks is, despite the performance not being very clear or exact [7]. Niu used the linear probability model to predict and analyze the operational risks of banks [8]. The results show that, using the linear probability model, most of the bankrupt banks can be successfully predicted within one to two years before the bankruptcy of banks, but the accuracy of the prediction results over three years is not significant. Shukla and Nanda analyzed the supervision and management principles of P2P peer-to-peer lending [9]. After analyzing the development of P2P, the predictable risks are also analyzed. Credit risks, capital risks, and money laundering through the Internet are all predictable risks. Cross-sectional regression model was used. The abovementioned scholars' research basically focuses on the selection of method models and many prediction experiments, which has certain research reference value.

### 2.2. Research on Neural Network Model

ANN (artificial neural network) is an important mathematical model, which is similar to the structure of synapses in the brain and can be used for information processing. Some scholars have proposed various types of chaotic neural network models [10], for example, the chaotic neural network model proposed by Kim et al., which can associate memory patterns aperiodically. Feng et al. proposed using coupled chaotic oscillator as a single neuron to construct chaotic neural network model [11]. Chakraborty and Chakraborty used BPNN (BP neural network) to forecast short-term traffic flow [12] and compared it with traditional forecasting models, such as the model based on historical data, time series model, and simulation model, and they concluded that BPNN was better than other models. Chen et al. proposed using recurrent neural network to forecast short-term traffic flow [13].

ANN provides gentle variable prediction while fuzzy neural network predicts the fluctuation effect. Adede et al. proposed a new type of area-based crack detector with deformable module, which can be used to improve the detection accuracy of surface cracks by comparing different models [14]. Kocadagli and Langari put forward a fault diagnosis method of rolling bearings using an improved 2D LeNet-5 network, which adjusts the number and size of convolution kernels and performs batch normalization. Experiments show that the improved method has higher fault diagnosis accuracy and less training time [15]. Ayvaz et al. used BPNN to build a liquidity risk early warning model of commercial banks [16].

## 3. Methodology

### 3.1. Construction of GFR Early Warning Index System for Commercial Banks

Different from the concept of traditional finance, green finance puts the environmental interests on which human beings depend in the first place, and the financial industry should serve the environmental protection. Green finance is a new stage in China, and people have a limited understanding of it. Environmental protection should be achieved through the joint efforts of all members of society, so it is more important to make green finance deeply rooted in people's hearts. After the implementation of green finance, the green added value of commodities has increased, and our commodities can meet the sales standards of these countries, broaden the sales channels of enterprises, and improve their reputation and status in the same trade.

Capital is the blood of economic activities. To change the norms of economic activities, the banking industry, as the hub of social capital financing, must also make adjustments, unify the economic responsibility and social responsibility of enterprises, strive to promote ecological civilization, and establish a comprehensive, coordinated, and sustainable development pattern. Green credit can avoid environmental risks. China is in the middle stage of industrialization, and its industrial structure is dominated by the secondary industry, especially the heavy chemical industry, with obvious characteristics of large consumption of industrial resources and large pollution discharge. Developing green credit is also an urgent need to improve the national happiness index and build a beautiful China. Commercial banks are shouldering an important mission, speeding up the development of green credit and supporting green industries, which will better coordinate the relationship between economic and ecological development and national happiness.

Early detection of commercial GFR is a crucial component of banks' overall credit risk management. In actual practice, the post-loan inspection and supervision of bank credit loans is the primary tool used by banks to monitor how they are using loans. It is also a crucial step in helping banks identify and prevent loan risk losses in a timely manner. As a result, the information for risk early-warning indicators is primarily based on the various statistical data, statements and sound records that the inspected commercial banks routinely submit.

To realise the monitoring function of credit risk early warning, the first step is to establish a scientific and reasonable early-warning index system. The first indication of the scientificity of the early-warning index system is whether the chosen index system can reflect the changing characteristics of commercial banks' credit risks and reasonably predict potential risks. All indicators must be organically coordinated to form a system that is neither repetitive nor contradictory in order to establish an early warning and evaluation index system for credit risk. At the same time, the calculation and evaluation methods for indicators must be rational and based on science. Early warning will lose its relevance if it cannot be delivered in advance to provide management the time to take appropriate action to reduce risks. In short, the criteria of comprehensive and scientific index content, predictability, pertinence, and operability should be followed in the development of credit risk early warning index systems.

Investment has the characteristics of short-term liquidity. The average debt term of Chinese banks is only about half a year, and the capital circulation cycle is short and high, which is the key for financial institutions to ensure value-added profits [17]. Therefore, the risk early warning index system of commercial banking system should be constructed at macro and micro levels. The schematic diagram of GFR index structure of commercial banks established in this paper is shown in Figure 1.

In the process of commercial banks' operation, customers' deposit and loan behaviors are completely random, so if the short-term credit supply accounts for a high proportion, it will bring additional risk burden to the banks' operation. The deterioration of commercial banks' assets will damage the capital movement of banks' credit ends, thus tightening monetary policy and raising market interest rates, threatening the stable development of financial markets.

PCA (principal component analysis) is to replace many original indexes with some small new quantitative index factors. Factor analysis is carried out by principal component extraction of common factors, and the main orthogonal factors of indicators are obtained, and the above variations are required to be explained.

According to the formula of factor analysis, set the following:

(1) $$\begin{array}{c} X_{i}=a_{i1}f_{1}+a_{i2}f_{2}+\cdots +a_{im}f_{m}+\varepsilon_{i}. \end{array}$$

The weight of the index *X*_*i*_ can be determined as follows:

(2) $$\begin{array}{c} \omega_{i}=\frac{\sum_{j=1}^{m}a_{ij}^{2}}{\sum_{i=1}^{n}\sum_{j=1}^{m}a_{ij}^{2}}, \end{array}$$

where *n* is the number of indicators, *m* is the number of factors in factor analysis, and *ω*_*i*_ is the weight of each indicator.

Initializing data, that is, dimensionless processing, that is, reducing the differences between index data, including the quantitative differences, followed by standardizing the processing matrix.

(3) $$\begin{array}{c} r_{ij}=\frac{\sum_{k=1}^{n}\left(x_{ki}-{\bar{x}}_{i}\right)\left(x_{kj}-{\bar{x}}_{j}\right)}{\sqrt{\sum_{k=1}^{n}{\left(x_{ki}-{\bar{x}}_{i}\right)}^{2}\sum_{k=1}^{n}{\left(x_{kj}-{\bar{x}}_{j}\right)}^{2}}}. \end{array}$$

External audit is an important external monitoring system of enterprises. Audit opinion refers to the opinions expressed by the auditor on whether the verification object meets the verification standards after completing the audit work.

### 3.2. Construction of Neural Network Model

The main promoter of green finance in China is the government, which promotes commercial banks, securities companies and insurance companies to develop green finance businesses such as green credit, green securities, and green insurance by issuing policies and regulations. Banks, securities, and insurance companies then conduct business with enterprises and consumers. The benefits of green finance will not appear immediately after its implementation, so it is difficult for commercial banks, securities, and insurance companies to obtain benefits in a short time, and risks will increase with the extension of time, so that financial institutions such as banks are reluctant to provide green products. Most green financial systems are principled, and regulatory measures lack feasibility and operability, and after obtaining financing funds, they continue to expand their original production lines, failing to make technical improvements and fulfill their environmental protection commitments, resulting in frequent environmental accidents and environmental violations.

The structure of the neural network is determined by the basic processing unit neurons and their interconnection methods. The basic processing unit of connection mechanism structure is often called neuron by analogy with neurophysiology. BPNN is a kind of neural network which is widely used in ANN [18]. It is considered to be the most suitable approximate relationship between analog input and output and has been widely used in the economic field. It is the most mature and widely used algorithm in ANN.

Figure 2 depicts the topology of the BPNN, a multilayer forward neural network with an error backpropagation learning mechanism. There are three layers in this network model: an input layer (IL), an output layer (OL), and a hidden layer (HL) between the input and OL. Because they do not have a direct connection to the outside world, there may be single-layer or multilayer HL.

In the BP network model, the basis function of neurons is linear, and its function form is as follows:

(4) $$\begin{array}{c} v=\overset{n}{\underset{j=1}{\sum }}w_{j}x_{j}-\theta =xw-\theta . \end{array}$$

The weight correction approach significantly affects the network performance in the first three-layer network algorithm. Here, the strategy described below is used:

(5) $$\begin{array}{c} w_{jh}\left(t+1\right)=w_{jh}\left(t\right)-\eta \frac{\partial E}{\partial w_{jh}}+\partial \left(w_{jh}\left(t\right)-w_{jh}\left(t-1\right)\right),\\ w_{hi}\left(t+1\right)=w_{hi}\left(t\right)-\eta \frac{\partial E}{\partial w_{hi}}+\partial \left(w_{hi}\left(t\right)-w_{hi}\left(t-1\right)\right). \end{array}$$

The structure of BPNN is simple, taking into account the convergence and accuracy of network training and avoiding the complicated description of internal rules of problems. These characteristics are suitable for solving the problems of many indicators and nonlinear correlation among indicators in GFR early warning model of commercial banks.

GFR is a double-edged sword. On the one hand, the function of the risk-endangering eco-environmental protection project has brought down the performance of ecological construction and protection and governance, and it is difficult to fundamentally solve the actual harm caused by the ecological environment crisis to the public. On the other hand, risks also damage the benefits of green investment and financing entities (including financial institutions and enterprises). Credit risk assessment and early warning of commercial banks is a very complicated system. The simple credit risk scoring model cannot describe this relationship well, and the processing results are quite different from the actual situation. In view of this situation, and in order to understand the operability in risk assessment and early warning of commercial banks in China, this paper constructs a GFR early warning model suitable for commercial banks by comprehensively applying ANN technology according to the concrete reality of our country.

In this paper, the forward three-layer BPNN technology is used to establish a real-time warning model of commercial banks' GFR. IL to HL adopts Sigmoid function, while HL to OL adopts linear function Purelin function. See Figure 3 for the specific modeling process.

Different GFR index systems of commercial banks correspond to different network models and also form different IL numbers, and the IL numbers are equal to the risk index numbers. To make the input data in the unsaturated region of Sigmoid function as far as possible, the sample data should be normalized according to the following formula:

(6) $$\begin{array}{c} x_{t}^{\prime }=\frac{x_{t}-x_{\min}}{x_{\max}-x_{\min}}, \end{array}$$

where *x*_max_, *x*_min_ represents the maximum and minimum values of the input sample data, *x*_*t*_ is the actual input original sample data, and *x*_*t*_′ is the normalized value. In this way, the input data will not fall into the saturation region of Sigmoid function, and the original characteristics of the data will not be changed.

We need to do the antinormalization operation again. The antinormalization formula is follows:

(7) $$\begin{array}{c} p=\frac{1}{2}\left(pn+1\right)\left(\max p-\min p\right)+\min p. \end{array}$$

In the above formula, max*p*, min*p* is the maximum value and minimum value in the sample data, *p* is the original sample data, and *pn* is the normalized value.

The parameter design is crucial for neural network application. The network can only converge rapidly and effectively and reach the specific error range by choosing the parameters right. A higher learning rate will typically cause the network to become unstable. It will begin to diverge too little if the error range is not reached, which will result in a prolonged training period, sluggish convergence, and the necessary error [19]. It is important to select the initial weight and threshold value sensibly in order to minimise the mistake. If it is too big, it is simple to enter the saturation area, which would terminate the network training. To increase the network's training pace, it is typically used as a random number uniformly distributed between [−1, 1].

When applying neural network method to model and solve practical problems, an important content is to determine the number of HL nodes. However, until now, based on a large number of foreign scientific research achievements, relevant scholars have summed up an empirical formula for this problem:

(8) $$\begin{array}{c} x\leq \sqrt{m\left(n+k\right)}+1. \end{array}$$

The number of HL nodes is represented by *x*, where *m* is the number of IL nodes, *n* represents the number of OL nodes, and *k* ∈ [2, 6]. According to the above empirical formula, the upper limit of the number of intermediate nodes in this model is 15. On this basis, according to the previous construction method, the model errors are compared, and the number of HL nodes is finally determined to be 11.

The error must be controlled within a reasonable range. First of all, the signal should be transmitted in OL. This error signal will propagate backward, correct the data along the familiar route, and determine a reasonable error threshold at the same time. The weight correction formula of hidden nodes is as follows:

(9) $$\begin{array}{c} {\delta_{i}}^{\prime }=f^{\prime }\left({\text{net}}_{k}\right)\underset{t}{\sum }\delta_{t}U_{jt}. \end{array}$$

Adjust the weight of the nodes, determine the appropriate threshold, and reduce the error so that the output of neurons is consistent with the target value.

## 4. Experiment and Results

The mapminmax function is used to normalize the acquired data so that all sample values fall within the range [0, 1], and the OL number is then calculated using the normalized data. The OL number is calculated using the error square sum of the neural network's actual and expected outputs as well as the number of training steps.  Table 1 and Figure 4 present the test findings. After comparative analysis, the OL number is 11 since there are few training steps and a tiny total of squared training errors.

Ten groups of input sample data are input into BPNN, and the corresponding output values of BPNN are obtained. Comparing the output result of expert comprehensive evaluation with the output value of BPNN, it is found that the error between them is not greater than the predetermined error. The data in Table 2 and Figure 5 show the training convergence process of these 10 groups of samples in the experiment. The results show that a well-trained BPNN evaluation model has been formed.

The probability of default refers to the possibility that the borrower cannot repay the loan principal and interest or fulfill the relevant obligations according to the contract requirements in a certain period of time in the future. According to the foregoing, the GFR real-time early warning model based on BPNN can model based on data and automatically generate fuzzy rules and adjust membership functions without expert experience. However, when an initial system is set up for training, the types of membership functions, the number of membership functions, and the training times are all to be determined.

The data of 100 commercial banks are trained, three parameters are randomly selected, and Gaussian membership function is adopted. The number of two membership degrees is 10 and 3, respectively, and the number of training times is 500. During the training process, the change trend of training times and RMSE (root mean square error) is shown in Figure 6.

It can be seen that RMSE is 0.0076 when the training times are 160. With 500 training times, RMSE is 0.0086. The difference between the two is only 0.001, but the workload of the latter is obviously much larger for computers. Therefore, the number of training times is not as much as possible, but the accuracy and the amount of calculation should be considered together. Therefore, the training times of the system constructed in this paper are 160.

Through the analysis of the above data, we can get that if we want to make effective use of BPNN, we need to use orthogonal design method, so that all parameters can be more reasonable. Compared with the early warning results of the existing neural network model, the multilevel index system is used as the input of the network, which makes the model more scientific. At the same time, it is not difficult to find out by comparing the dispersion degree of prewarning results. Taking the index system as input can increase the accuracy of early warning.  Figure 7 shows the trends of optimal learning rate.

The number of OL significantly affects how quickly the network converges. The performance of the network does not increase with the number of HL neurons. This experiment demonstrates the benefit of having more OL. Numerous trials should be conducted to determine the precise amount of OL. The following types of errors are defined in this document with regard to the loss of the judgement outcome to the bank: the first type of mistakes misread samples with low alarm levels as being high alarm levels, whereas the second type of mistakes misjudges samples with high alarm levels as being low alert levels.  Figure 8 displays the outcomes of testing 50 test samples using the previously trained network.

It can be seen that the test result of this method is greatly improved compared with that of the traditional method, and the correct rate is increased from 81.27% to 94.38%. At the same time, there are fewer cases of making the second kind of mistakes. It can be seen that this method is better than the traditional method and obviously improves the adaptability and robustness of the algorithm.

In the face of the unique development situation of green finance, green credit, bonds, green stock index and development funds can be adopted to promote the greening of the financial system. The government can also introduce relevant green financial policies, give support and match resources in the field of international cooperation, diversify financing, and broaden channels. At the same time, it is also possible to take the form of “equity+creditor's rights” investment to dominate the financing form of the new district. According to the specific industrial characteristics, draw lessons from the relevant rules and standards of developed countries to formulate the green financial legal system, and evaluate and measure the financial supervision, so as to achieve the goal of standardized operation of financial environmental risk rating.

Green development, circular development and low-carbon development are the fundamental ways to improve the ecological environment, alleviate the shortage of resources and cope with climate change, and the fundamental measures to ensure people's ecological safety, production safety and life safety. As for the evaluation and investigation of green credit, it is a comprehensive and professional field. Appraisers should not only have a solid financial and financial knowledge reserve but also learn the knowledge of environmental science, have a certain research and grasp of the evaluation standards and guidelines, and at the same time, follow the national policy directions in time, so as to learn from experience, reserve talents, cultivate high-quality professional talents, and be in line with international standards.

The early warning system must continuously update the information and implement real-time information collecting, according to the fundamental concept of information theory. Therefore, the bank supervisory information network needs to be swiftly constructed to assure the credit risk early warning system's effectiveness. Implement thorough risk assessment and management, raise credit risk management's scientific theoretical level, anticipate credit risks using science, and track and monitor loans item by item. Accurately comprehend the structure, analysis, and quality of the total amount of credit assets and identify and promptly address the illegal activities of financial institutions and their branches, in order for banks to have a more thorough and reliable foundation for the supervision of large loan management, large loan management, and off-site surveillance of financial institutions and to increase the level of financial regulation and supervision. Personnel responsible for risk warnings should have a thorough understanding of the credit industry as well as good analytical skills. Improve the idea of risk management, keep up with changes in the industrial knowledge base, become proficient in a wide range of cutting-edge tools and methodologies for analysis, and raise the bar for risk early warning analysis.

## 5. Conclusions

Investment in green finance eco-environmental protection projects has clear social advantages, but the risks and rewards are unclear. As a result, the standard of macro-prudential supervision for green financial projects is low, and there are several gaps in micro-prudential supervision, which is also a crucial element in determining the risk associated with using green financial practices. It is the backbone of the contemporary financial system, and risk management is one of its primary tenets. Early warning refers to a warning that is sent ahead of time, advising individuals to pay attention to the imbalanced condition, abrupt occurrences, and disordered structure that will manifest during system operation and to take prompt action to move the system into a new structural state. Given that GFR early warning currently imperfects both domestically and internationally, a new GFR early warning model for commercial banks is created using a neural network model, and the current state of green finance in commercial banks is examined using reliable data from various indicators of the system. The test outcome of this method is significantly better than the previous way, according to the data, and the accuracy rate has grown from 81.27% to 94.38%. It is clear that this strategy outperforms the conventional approach and enhances the algorithm's robustness and adaptability.

## Figures and Tables

**Figure 1:** Schematic diagram of GFR index structure of commercial banks.

**Figure 2:** BPNN structure.

**Figure 3:** GFR early warning system model of BPNN commercial bank.

**Figure 4:** Network training error.

**Figure 5:** Comparison chart of output values.

**Figure 6:** Training times and the changing trend of RMSE.

**Figure 7:** Optimal learning rate chart.

**Figure 8:** Algorithm test results.

**Table 1:** Selection of OL number.

OL number	Network training error	Training steps
1	0.2673	99
2	0.1709	63
3	0.254	70
4	0.2898	113
5	0.2772	64
6	0.2902	112
7	0.2767	91
8	0.2061	86
9	0.138	135
10	0.2557	128
11	0.0504	95
12	0.3032	48
13	0.2831	78
14	0.2516	90
15	0.2128	114

**Table 2:** Comparison between comprehensive evaluation by experts and actual output value of corresponding BPNN.

Sample	Expected output	Actual output
1	2.0203	2.0207
2	2.0206	2.0202
3	2.0203	2.0207
4	2.0201	2.021
5	2.0205	2.0204
6	2.0204	2.0206
7	2.0205	2.0202
8	2.0203	2.02
9	2.0201	2.021
10	2.0208	2.02

## Data Availability

The data used to support the findings of this study are available from the corresponding author upon request.
